# Linking Prioritized Occupational Performance in Patients Undergoing Spasticity-Correcting Upper Limb Surgery to the International Classification of Functioning, Disability, and Health

**DOI:** 10.1155/2022/8741660

**Published:** 2022-10-14

**Authors:** Therese Ramström, Johanna Wangdell, Carina Reinholdt, Lina Bunketorp-Käll

**Affiliations:** ^1^Centre for Advanced Reconstruction of Extremities, Sahlgrenska University Hospital/Mölndal, Häraldsgatan 16, 431 30 Mölndal, Sweden; ^2^Institute of Clinical Sciences, Department of Hand Surgery at Sahlgrenska Academy, University of Gothenburg, Göteborgsvägen 31, 431 80 Mölndal, Sweden; ^3^Institute of Neuroscience and Physiology, Department of Health and Rehabilitation, Sahlgrenska Academy, University of Gothenburg, Box 430, 405 30 Gothenburg, Sweden

## Abstract

**Background:**

Spasticity is generally caused by damage to the spinal cord or the areas of the brain that controls movements, which poses significant limitations in occupational tasks.

**Objectives:**

The aims of the study were to (I) describe prioritized occupational performance problems (POPP) among patients who underwent upper limb spasticity-correcting surgery and map them to the International Classification of Function, Disability, and Health (ICF); (II) assess outcomes postsurgery; (III) assess whether the results are influenced by the diagnosis, gender, and residual muscle function; and (IV) assess correlation between changes in COPM and gains in grasp ability and grip strength.

**Methods:**

In this retrospective study, assessments occurred pre- and postsurgery, including the Canadian Occupational Performance Measure (COPM), grip strength, and grasp ability. POPP were transformed to prioritized occupational performance goals (POPG) during subsequent rehabilitation.

**Results:**

60 patients with a history of spinal cord injury (SCI) (*n* = 42; 59%), stroke (*n* = 25; 34%), traumatic brain injury (TBI) (*n* = 4; 6%), and reason unknown (*n* = 1; 1%) were included, with a mean age of 57 (±13) years. Of those, 11 had bilateral surgery, generating 71 COPM forms and 320 POPG. The POPG were mapped to the ICF activity and participation chapter, most often to self-care (*n* = 131; 41%), domestic life (*n* = 68; 21%), and mobility (*n* = 58; 18%). COPM scores were significantly increased postsurgery, irrespective of diagnosis, gender, and muscle function. No clear correlation between COPM improvement and hand function gains was shown.

**Conclusion:**

Patients who underwent spasticity-correcting upper limb surgery identified difficulties with a wide range of occupational tasks that they considered as important to regain. Treatment-induced gains in occupational performance were significant but had no clear correlation with gains in grasp ability and hand strength. Independent of diagnosis, gender, and residual muscle function, it seems important to address the activity- and participation-specific aspects in the assessment and rehabilitation of patients.

## 1. Introduction

The ability to perform everyday occupations is essential to human well-being and an important part of one's identity [1]. Enhancement of occupational performance is therefore a core construct in rehabilitation and especially in occupational therapy. Various injury and disease-related symptoms cause difficulties in the occupational capacity of patients. Spasticity is a common secondary complication to central nervous system (CNS) injuries. Spasticity often limits upper limb (UL) movements and therefore interferes with daily life activities [2]. Muscle weakness or paralysis may further hamper the ability to engage in daily activities [3]. Hand grip dynamometry is commonly used to measure grip strength, which in general can be interpreted as an indicator of overall UL strength [4]. Cut-off values for the grip strength needed to manage different tasks, especially heavy tasks, are available [5]. Grasp ability is another common measure to evaluate UL capacity. Research findings have demonstrated low correlations between grip strength and dexterity, as well as between dexterity and grasp ability [6]. Whether grip strength and grasp ability could be linked to occupational performance in a population with UL spasticity is yet unknown.

The clinical presentation of individuals with spasticity is heterogenous, which is why clinical guidelines recommend spasticity management to follow a multidimensional approach [7]. Spasticity management is also said to benefit from a client-centered and goal-oriented approach [7]. Due to the heterogeneity of spasticity-related disorders, the treatment goals are often diverse and depend on the ambition, priorities, and residual muscle function of the individual. This diversity in interventional goal settings makes it a challenge to find appropriate outcome measures to be used on a group level. Individualized goal setting makes patients more likely to engage in their rehabilitation [8]. Goal setting is also helpful for clinicians when tailoring rehabilitation to the specific needs of individuals. Clear goals enhance motivation and lead to better outcomes, and they are also effective for understanding and changing human behavior [9]. One purposeful measure that can help identify patients' performance problems is the Canadian Occupational Performance Measure (COPM) [10]. The COPM tool is based on semistructured interviews. COPM uses a client-centered approach to help patients identify prioritized occupational performance problems (POPP), that is, occupational issues of particular relevance to them. POPP identified with COPM can be classified using the International Classification of Function, Disability, and Health (ICF) [11]. The ICF model uses a shared language to classify the impact of diseases across different health or health-related domains. In the ICF, activity and participation are treated as 1 component, yet they have different definitions. ICF defines activity as the execution of a task or action by an individual and participation as an individual's involvement in life situations [11]. Due to the heterogeneity of individuals suffering from UL spasticity, an individualized client-centered outcome measure such as COPM could be particularly helpful. To investigate this further, we designed the present study with the aim to (I) describe POPP that individuals who underwent UL spasticity-correcting surgery considered the most important and map these problems to the ICF; (II) assess the perceived level of performance and satisfaction 6–12 months after surgery; (III) assess whether results are influenced by diagnosis, gender, and residual muscle function; and (IV) assess the correlation between gains in performance and satisfaction as an outcome of surgery and gains in grasp ability and grip strength.

## 2. Method

### 2.1. Study Design and Setting

This is a retrospective mapping study that involves secondary analyses of data collected in previous studies [12, 13]. Applications were sent to the Swedish Ethical Review Authority for both studies (Dnr 2019-05162 and 407-16). Since the ethics committee declared the studies were considered part of clinical work and that data was gathered as part of routine care, ethical approvals for the studies were not required, and consent was therefore waived. The study was conducted in accordance with the Helsinki Declaration. The study participants are patients who underwent surgery to lessen spasticity-occupational problems in the UL. All surgeries were performed at one center. The data was collected the day before surgery (baseline) and 6 and 12 months after surgery (follow-up).

### 2.2. Surgical Procedure and Subsequent Rehabilitation

The spasticity-correcting surgical procedures included primarily tendon lengthening and, to a lesser extent, release of muscles, and they have previously been described in detail [12, 13]. A very sound judgement of appropriateness was made in every single case using a team-based approach, and the surgical intervention was always preceded by detailed information about what to expect from the procedure. Prior to surgery, patients were stratified to receive a regimen-specific rehabilitation (high-, low-, or nonfunctioning regimen; HFR, LFR, NFR) depending on their remaining volitional UL muscle function [13]. Patients allocated to the HFR were expected to improve volitional muscle control after surgery; hence, their ability to use the affected arm in unimanual activity was expected to increase. Patients allocated to the LFR were expected to increase their ability to use the affected arm in bimanual UL activity. In the NFR, the goal was mainly to facilitate personal hygiene activities and resting position of the UL. Three weeks after surgery, patients returned to the center for follow-up assessments and an inpatient stay to commence activity-based training. The training was individualized and based on the specific POPP that were documented by means of COPM prior to surgery. In the Appendix, the surgical technique and rehabilitation are briefly described.

### 2.3. Participants

The patients were consecutively recruited according to the following inclusion criteria: (I) underwent spasticity-correcting surgery between the years 2015 and 2020, (II) treated according to HFR or LFR, (III) had COPM data collected on one or several occasions, and (IV) having spasticity problems in the UL due to CNS injury. Spasticity was measured with Modified Ashworth Scale [14]. An exclusion criterion was (I) treated according to NFR and thus was not expected to achieve any activity performance gains.

## 3. Data Collection

### 3.1. Measures

A patient's own perception of occupational problems that he or she encountered due to UL spasticity was measured with COPM. The COPM is an individualized assessment tool designed for measuring changes in occupational performance of individuals receiving occupational therapy [10]. The COPM is administered through a semistructured interview where the person reports those daily activities that he/she perceives as difficult to perform. In line with this study, we asked patients to identify occupational activities commonly performed with the UL. From among these, the patients were asked to select the five most important activities. Commonly, the selected activities are then used to formulate the personal treatment goals. To ensure that patients' prioritized goals were realistic and achievable, the patients underwent a thorough clinical examination and were given extensive information about the surgical procedure and subsequent rehabilitation. According to the manual, the ratings are summed and presented as mean scores of performance and satisfaction [10]. Higher ratings indicate greater performance and increased satisfaction. After an intervention, the performance and satisfaction with the performance of the targeted POPP are again rated on the scale. When used as an outcome measure, each individual rating of performance and satisfaction with performance is summarized, and mean values, representing overall scores in performance and satisfaction with performance, are calculated. According to the COPM manual, a change in mean score of at least 2 represents a minimal clinically important difference (MCID) [10]. The COPM instrument is shown to have good validity and good test-retest reliability, and it is sensitive to change in an adult population [10].

Maximum handgrip strength was measured with a hydraulic hand dynamometer (JAMAR® 5030J1, Sammons Preston Rolyan, USA) [15]. The participant was seated in a standard position, and the maximum value of three attempts was used for analysis.

The ability to grasp, move, and release objects was measured using the Grasp and Release Test (GRT). The GRT is a timed test developed for measuring grip ability in individuals with tetraplegia [16]. In the GRT, the patient is to pick up, move, and release six objects of varying sizes, weights, and textures using a palmar or lateral grasp. The number of items successfully transferred in 30 seconds is recorded [16].

### 3.2. Data Analysis

Demographics and baseline characteristics were summarized using descriptive statistics. The POPP identified with COPM were mapped according to the ICF [11] in line with guidelines developed by Cieza et al. [17, 18]. In the context of this study, these POPP are referred to as prioritized occupational performance goals (POPG). Data was analyzed for the study group as a whole, as well as for subgroups of patients with respect to diagnosis, gender, and treatment regimen. Missing data at 12 months was replaced with the previous observation at 6 months. The Wilcoxon signed rank test was used to analyze changes in outcome measures. The Mann-Whitney *U* test was used to assess group differences with respect to changes in outcome measures. All tests of significance were 2-sided; *p* < 0.05 was considered statistically significant. In line with previous findings [10], a change ≥ 2 was considered an MCID. The Spearman correlation was used to assess the relation between gains in perceived performance and satisfaction measured with COPM as a result of surgery and treatment-induced gains in grasp ability and grip strength. The Spearman correlation results were interpreted according to an often quoted rule of thumb: 0.90–1.00, very high; 0.70–0.90, high; 0.50–0.70, moderate; 0.30–0.50, low; and 0.00–0.30, little or none [19].

## 4. Results

A total of 60 patients were included in the study. Of these 60 individuals, 11 had undergone surgery on both the right and left arm on different occasions, which means that the total number of surgeries amounted to 71 (Figure 1). The mean age was 57 years with an age range of 24–79 years, and there were 42 men (59%) and 29 women (41%). The mean time elapsed since injury was 8.5 years [1–35]. The spasticity was a consequence following spinal cord injury (SCI) (*n* = 42; 59%), stroke (*n* = 25; 34%), TBI (*n* = 4; 6%), or a reason unknown (*n* = 1; 1%). The patients were stratified to receive HFR (*n* = 34; 48%) or LFR (*n* = 37; 52%). Demographics, clinical characteristics, and stratification based on treatment regimen and diagnosis are presented in Table 1.

### 4.1. Mapping of Prioritized Occupational Performance Goals to the ICF

Altogether, patients identified 320 POPG that were considered of great relevance for them. All POPG were classified as belonging to the activity and participation component of ICF, often related to self-care (*N* = 131; 41%), followed by domestic life (*N* = 68; 21%), mobility (*N* = 58; 18%), communication (*N* = 31; 9.7%), social and civic life (*N* = 8; 2.5%), interpersonal interactions and relationships (*N* = 19; 5.9%), and major life areas (*N* = 4; 1.2%). The mapping of goals according to the ICF categories is presented in Table 2 and Figure 2. Self-care was the most frequently targeted ICF domain, independent of diagnosis, gender, and treatment regimen. In Figure 2, the mapping of goals is stratified with respect to diagnosis, gender, and treatment regimen.

The five most frequent POPG, as classified on the more specific domain level, were preparing meals (15%), dressing (13.4%), eating (13.9%), recreation and leisure (5.9%), and drinking (5.6%).

### 4.2. Treatment-Induced Changes in COPM

The mean COPM-P score for the whole study group increased by 2.5 ± 2.9, from 2.3 ± 1.1 at baseline to 4.8 ± 2.0 at the 12-month follow-up (*p* = 0.001), thus exceeding the predefined MCID of 2.0 [10]. Corresponding figures for the groups stratified on the basis of diagnosis, gender, and treatment regimen yielded equivalent results with no significant difference with respect to changes in COPM-P scores between the stratified groups. Patients with SCI (*n* = 36) and stroke (*n* = 22) had a mean COPM-P increase of 2.4 ± 1.8 (*p* = 0.001) and 2.5 ± 1.7 (*p* = 0.001), respectively, with no significant difference between groups (*p* = 0.745). When the analyses were split by gender, the male patients (*n* = 45) had a mean COPM-P increase of 2.5 ± 1.9 (*p* = 0.001) and women had 2.7 ± 1.6 (*p* = 0.001), with no significant difference between genders (*p* = 0.725). Patients in the HFR group (*n* = 29) had a mean COPM-P increase of 2.8 ± 2.2 (*p* = 0.001), whereas the corresponding increase for the patients in the LFR group (*n* = 31) was 2.2 ± 1.4 (*p* = 0.000), with no significant difference between groups (*p* = 0.205). Mean COPM scores at baseline and follow-up in the whole study group and divided in subgroups are presented in Figure 3.

Of the 320 POPG identified by participants, 134 (42%) were assigned score 1 at baseline, meaning they were perceived as impossible to perform by patients. These 134 goals were mapped to the ICF as follows: self-care (*n* = 60; 44.8%), domestic life (*n* = 26; 19.4%), mobility (*n* = 20; 14.9%), community, social, and civic life (*n* = 13; 9.7%), communication (*n* = 10; 7.5%), interpersonal interactions and relationship (*n* = 3; 2.2%), and major life areas (*n* = 2; 1.5%). The COPM-P ratings at 12 months showed that 89 of the 134 goals (66%) had become possible to perform as a result of the treatment; of these, 45 (33.5%) were assigned performance scores of 5 or higher.  Table 3 shows changes in COPM mean scores from pre- to postsurgery.

In line with the results of the COPM-P analyses, there was a significant increase in COPM-S mean score (2.7 ± 2.1; *p* = 0.001) from pre- to postsurgery for the whole study group (*n* = 59).

Further analyses of the SCI (*n* = 36) and stroke (*n* = 21) subgroups revealed similar increases of 2.4 ± 2.1 (*p* = 0.001) and 3.0 ± 1.7 (*p* = 0.001), respectively. Male (*n* = 44) and female (*n* = 15) patients had mean COPM-S increases of 2.6 ± 2.2 (*p* = 0.001) and 3.1 ± 1.6 (*p* = 0.001), respectively. Corresponding figures for the HFR (*n* = 29) and LFR (*n* = 30) subgroups were 2.9 ± 2.6 (*p* = 0.001) and 2.6 ± 1.5 (*p* = 0.001), respectively. In the stratified subgroup analyses (diagnosis, gender, and treatment regimen), no significance between group differences with respect to the change in COPM-S mean scores was shown (*p* = 0.263, 0.440, and 0.490, diagnosis, sex, and regimen, respectively).

### 4.3. Correlation Analyses

The results of the correlational analyses between changes in COPM-P mean scores pre- to postsurgery and gains in grasp ability showed little or no correlation (*r*_*s*_ = 0.297; *p* = 0.025), whereas no significant relationship between change in COPM scores and grip strength was shown. There was a strong significant correlation between the changes in COPM-P and COPM-S scores. See Table 4 for details.

## 5. Discussion

The findings of the present mapping study demonstrate that POPG specified by patients with spasticity-related disorders who underwent spasticity-correcting surgery covered a wide range of activities. Independent of diagnosis, gender, and residual UL volitional muscle function prior to surgery, POPG were often related to self-care activities. The problems identified by the patients in this study could be linked to seven different ICF domains, highlighting the diversity of occupational problems that individuals with UL spasticity commonly experience. The results are in line with previous qualitative findings of how spasticity commonly interferes with activities of daily living [20, 21]. Although the identified problems in the present study were mapped onto several ICF domains, the majority were related to self-care, domestic life, and mobility. Independence has previously been reported as a primary goal, both in the context of in-patient rehabilitation and in the community [22]. A similar distribution of occupational problems has been demonstrated for individuals suffering from SCI [22, 23]. The fact that self-care activities and mobility are essential for independence in daily life could be the reason for those activities being most commonly prioritized by patients in both the present and previous studies.

To the best of our knowledge, this is the first study to report and classify POPG according to ICF in a cohort of patients stratified in groups based on diagnosis, gender, and severity of UL impairment. Previous reports exist on the same theme but involve patients with disabling spasticity who are receiving botulinum toxin treatment [24, 25] or are limited to patients with SCI only [26]. COPM has previously been used to demonstrate positive POPG outcomes in a mixed population undergoing spasticity-correcting surgery [12] and with patients split into regimens [13]. These reports, however, have their main focus on outcome assessment and do not primarily aim to map the POPG set by patients receiving surgical treatment for disabling UL spasticity.

The fact that some patients with a history of stroke identified goals in the communication domain (11.5%) may be explained by cognitive sequelae such as aphasia being more frequent among stroke survivors, compared to individuals with SCI. The proportion of patients with SCIs who prioritized goals related to mobility was rather high (24.5%), whereas somewhat fewer patients in the stroke group (11.5%) selected such goals. The transfers were not identified in this study, but it is likely that the proportion of wheelchair users is higher in the SCI group, which can explain this difference. Individuals with SCI commonly targeted goals relating to self-care activities (43.3%), which is not very surprising given that regaining hand function is considered the foremost priority among individuals living with debilitating consequences that follow SCIs [27]. Moreover, for individuals in the stroke group, activities within the self-care domain were frequently targeted, as were home-related activities such as preparing meals, doing housework, and caring for household objects. Occupational performance problems within domestic life were also considered important to regain among individuals with SCI. Since rehabilitative interventions often have their primary focus on self-care activities, attention should be paid to the fact that activities such as cooking and housework may be of similar importance to patients and should be addressed in rehabilitative situations. Both women and men primarily considered occupational performance tasks within the self-care domain as the most important to regain. The second most important problem chosen among males was mobility related, whereas the second most common POPG identified by females were related to domestic life. The surgery brought about a significant improvement in patients' perceived occupational performance as measured by COPM, irrespective of diagnosis, gender, and regimen.

Improvement in participation is proposed to be the most valued outcome for patients [28]. The ICF [11] proposes four different ways of separating the nine domains included in the activity and participation domain. Some authors suggest that participation involves a variety of tasks; others mean that it requires a social context [29]. Self-care is often linked to activity while mobility and domestic life often are linked to participation [29]. Eating is however an activity linked to self-care that can be an activity itself or related to a social context. For some people, the goal can be the act of eating, whereas for others, the importance lays in the social context of eating. To distinguish between activity and participation was therefore not possible in this retrospective study.

Patients in the present study were allocated to receive a high- or low-functioning treatment regimen depending on the degree of remaining UL muscle function. For patients with high residual muscle function, surgery aimed to bring about gains in the patients' ability to use the affected arm in unimanual activities. This may be the reason for those patients selecting self-care activities often accomplished with one arm, such as combing hair, brushing teeth, grasping, and drinking from glasses. In line with our previous findings on spasticity-correcting surgery [13], showing that our patients with SCI often have sufficient residual volitional muscle function for them to be allocated to receive HFR, the proportion of patients with SCI was higher in that group compared to patients with stroke. For individuals with stroke, spastic hemiplegia commonly enables them to receive LFR, with the aim of increasing the ability to use the affected arm in bimanual activities.

The results of the present study are in agreement with previous findings in a cohort of patients with SCI [26], demonstrating that 34% of the prioritized occupational performance goals could be mapped to the self-care domain, followed by domestic life (19%), mobility (16%), and the communication domain (12%). Since the previous study by Wangdell et al. [26] included only patients with SCI, only comparisons with our SCI subgroup are feasible. For the SCI group in the present study, the changes in mean COPM-P and COPM-S scores were 2.4 and 2.4, respectively, compared to 2.7 and 3.2 in the Wangdell SCI cohort. At the time of the previous study, patients were not split into different treatment regimens (based on residual muscle function), but they might have consisted of patients with a larger degree of remaining volitional muscle function, which in turn increases the probability of achieving beneficial gains from surgery. This highlights the importance of assessing the levels of remaining muscle function in relation to the expected gains to be achieved by surgery to be able to judge the transferability of the results to another setting or group of individuals.

Grip strength has in previous studies been suggested to serve as a predictor of overall hand function, and it could aid in predicting mobility, personal care, and disability later in life [4]. Furthermore, Bohannon has demonstrated that overall strength and UL function are associated with grip strength [4] and further concludes that grip strength can be recommended as a standalone measurement [4]. Previous findings have demonstrated that recovery of grip strength could be linked to overall hand function and activities [30]. In the present study, however, gains in grasp ability and grip strength were not or were weakly correlated with the changes in COPM mean scores. These weak or absent correlations are in line with the findings by Wangdell and Friden [31], demonstrating no significant correlation between outcomes in body function and perceived performance of the prioritized goals after reconstructive hand surgery in tetraplegia. In line with the findings in the present study and previous findings [32], grip strength could not be recommended as a standalone measurement to mirror the motor control of the hand for disabled individuals. Daily activities are complex and conducted in a dynamic interaction between the individual's personal factors, the performed activity, and the environment. The lack of correlation between activity performance, satisfaction, grasp ability, and hand strength indicates the importance of addressing activity-specific aspects in the rehabilitation of patients. Besides, to transform gains in body function to gains relating to activity and participation in daily living, task-specific training is beneficial [33].

The importance of identifying relevant patient-centered goals in rehabilitation practices and interventions has previously been highlighted [8]. Assisting in setting appropriate goals may facilitate communication between patients and clinicians. The use of free goal setting is more time demanding and has raised concerns about lack of standardization and comparability [34]. Standardized measures that have a set of predefined goals to be rated by patients provide a more streamlined way of identifying goals that are of importance for patients and make comparisons more appropriate. However, Patient Reported Outcome Measures (PROMs) with predefined activities can involve activities of no importance for the individual. Another way to streamline goal-setting procedures is to use a goal bank as a guide to assist with goal setting [24].

## 6. Limitations

There are some limitations that must be considered when interpreting the results of this study. Due to the retrospective study design, some patients had incomplete follow-up data and could not be included in the analyses. Furthermore, the study setting was limited to one single center, which limits the generalizability. The fact that the therapy providers and assessors in the present study were the same could potentially have biased the results. Since the COPM targets activity and participation limitations and not body function and structure, the goals specified by patients are purely related to the activity and participation component. In this study, we have not separated the ICF component activity and participation into different categories. We can therefore not draw conclusion if goals relating to activities or participation are influenced by diagnosis, sex, or regimen. Concerns about the absence of standardization in the individual goal setting, such as when using COPM, have been raised since it may limit comparability across different populations and settings [35].

## 7. Conclusion

The wide range of occupational problems that the patients in the present study considered important to regain prior to surgical treatment highlight the diversity of disablement that UL spasticity entails. A large majority of the identified problems were related to self-care, domestic activities, and mobility aspects, irrespective of diagnosis, gender, and treatment regimen. Thus, rehabilitation practices should address not only self-care activities but also activities such as cooking and housework tasks that may be of similar importance to patients, as well as communication for individuals with such problems. The surgery brought about significant improvement in patients' perceived occupational performance even though little or no correlation between patients' perceived gains in occupational performance and change in grasp ability and grip strength was shown. This highlights the importance to include outcome measures covering different ICF domains in treatments targeting UL performance. Finally, the findings of the present study could be used to inform patients about the potential benefits of spasticity-correcting surgery.

## Figures and Tables

**Figure 1:** Study flow. ICF = International Classification of Functioning, Disability, and Health; COPM = Canadian Occupational Performance Measure.

**Figure 2:** ICF mapping of occupational performance goals identified by the study population as a whole and split in diagnosis, sex and regimen. SCI = spinal cord injuries; HFR = high-functioning regimen; LFR = low-functioning regimen.

**Figure 3:** Mean Canadian Occupational Performance Measure scores at baseline and at the 12-month follow-up, presented as mean score, split in (a) all goals and ICF chapters COPM-P, (b) all goals and ICF chapters COPM-S, (c) study group as a whole, (d) diagnosis, (e) sex, and (f) treatment regimen. SCI = spinal cord injuries; HFR = high-functioning regimen; LFR = low-functioning regimen; Interpersonal interactions &… = interpersonal interactions and relationships; COPM-P = Canadian Occupational Performance Measure-Performance; COPM-S = Canadian Occupational Performance Measure-Satisfaction. ^∗^ indicates significant difference below 0.005, ^∗∗^ indicates significant difference below 0.001, and error bars indicate standard error means.

**Table 1:** Demographic and clinical characteristics of the study population as a whole and split in diagnosis, regimens, and sexes.

	Whole population	Split in diagnosis		Split in treatment regimen		Split in sexes	
	Total	SCI	Stroke	HFR	LFR	Female	Male
Patients (%)	71 (100)	42 (59)	24 (34)	34 (48)	37 (52)	19 (27)	52 (73)
Age mean (min–max)	57 (24–79)	57 (24–79)	59 (42–76)	55 (28–79)	60 (24–76)	53 (24-76)	59 (41-79)
Gender							
Women	19 (27)	6 (14)	10 (42)	6 (18)	13 (35)	19 (100)	0 (0)
Men	52 (73)	36 (86)	14 (58)	28 (82)	24 (65)	0(0)	52 (100)
Diagnosis							
SCI	42 (59.1)	42 (100)	0 (0)	25 (73.5)	17 (45.9)	6 (32)	36 (69)
Stroke	24 (33.8)	0 (0)	24 (100)	8 (23.5)	16 (43.2)	10 (53)	14 (27)
TBI	4 (5.6)	0 (0)	0 (0)	1 (2.9)	3 (8.1)	2 (10)	2 (4)
Other/unknown	1 (1.4)	0 (0)	0 (0)	0 (0)	1 (2.7)	1(5)	0 (0)
Regimen							
HFR	34 (48)	25 (59)	8 (33)	34 (100)	0 (0)	6 (32)	28 (54)
LFR	37 (52)	17 (40)	16 (67)	0 (0)	37 (100)	13 (68)	24 (46)
Time (years) between injury and surgery mean (min–max)	8 (1–35)	7 (1–30)	10 (1–32)	8 (1–35)	8 (1–26)	12 (1-30)	7 (1-35)

SCI = spinal cord injuries; HFR = high-functioning regimen; LFR = low-functioning regimen; Min = minimum; Max = maximum; TBI = traumatic brain injury.

**Table 2:** Mapping occupational performance goals according to the International Classification of Function, Disability, and Health (ICF) (*n* = 320).

ICF chapter	ICF domain	*N* (%)	Frequencies (percentage within chapter/total)
Communication		31 (9.7)	
	Receiving nonverbal messages		5 (16.1/1.6)
	Writing messages		11 (35.5/3.4)
	Using communication devices and techniques		15 (48.4/4.7)

Mobility		58 (18.1)	
	Changing basic body position		1 (1.7/1)
	Maintaining a body position		3 (5.2/.9)
	Transferring oneself		4 (6.9/1.3)
	Lifting and carrying objects		7 (12/2.2)
	Fine hand use		16 (27.6/5.0)
	Hand and arm use		4 (6.9/1.3)
	Walking		3 (5.2/.9)
	Moving around		2 (3.4/.6)
	Moving around using equipment		12 (20.7/3.8)
	Driving		6 (10.3/1.9)

Self-care		132 (41.3)	
	Washing oneself		11 (8.3/3.4)
	Caring for body parts		17 (12.9/5.3)
	Toileting		5 (3.8/1.6)
	Dressing		43 (32.6/13.4)
	Eating		38 (28.8/11.9)
	Drinking		18 (13.6/5.6)

Domestic life		68 (21.3)	
	Preparing meals		48 (70.6/15.0)
	Doing housework		15 (22.1/4.7)
	Caring for household objects		5 (7.3/1.6)

Interpersonal interactions and relationships		8 (2.5)
	Basic interpersonal interactions		8 (100/2.5)

Major life areas		4 (1.3)
	Remunerative employment		4 (100/1.3)

Community, social, and civic life		19 (5.9)
	Recreation and leisure		19 (100/5.9)

**Table 3:** Change in COPM performance and satisfaction from baseline to follow-up (12 months) dichotomized into groups based on degree of change.

		n	Negative change/no change ≤ 0	Positive change > 0 < 2	Clinically significant change ≥ 2
Whole group	Performance	60	3	22	35
	Satisfaction	59	6	16	37
SCI	Performance	36	2	14	20
	Satisfaction	36	6	9	21
Stroke	Performance	22	1	7	14
	Satisfaction	21	0	6	15
HFR	Performance	29	2	10	17
	Satisfaction	29	5	6	18
LFR	Performance	31	1	12	18
	Satisfaction	30	1	10	19

SCI = spinal cord injuries; HFR = high-functioning regimen; LFR = low-functioning regimen. Data dichotomized into (I) negative change or no change, difference ≤ 0; (II) positive change, between +0.10; and (III) +1.99 and clinically significant change, ≥2.

**Table 4:** Association between change in Canadian Occupational Performance Measure (COPM) scores and Grasp and Release Test (GRT) and between change in COPM scores and grip strength (JAMAR) from baseline to the 12-month follow-up.

	*n*	COPM-P		*n*	COPM-S	
		*r*_*S*_	*p*		*r*_*S*_	*p*
COPM-P	59			59	.855	*<.001*
COPM-S	59	.855	*<.001*	59		
GRT	57	.297	*.025*	56	.239	.076
Grip strength	48	.245	.093	48	.161	.274

*r*_*S*_ = Spearman correlation coefficient; COPM = Canadian Occupational Performance Measure; P = performance; S = satisfaction; GRT: Grasp and Release Test. Significant correlations are presented in italics.

## Data Availability

The data that support the findings of this study are available from the corresponding author, TR, upon reasonable request.

## Appendix

### A. Description of the Spasticity-Correcting Surgical Treatment and Subsequent Rehabilitation

#### A.1. Preoperative Assessments

Prior to surgery, all patients had tried conservative treatment. When the conservative approach consisting of physiotherapy, occupational therapy, orthosis, medication and/or botulinum toxin injections was not sufficiently effective, surgery was brought up as an alternative treatment option. Overall health parameters were consulted by an anesthesiologist and addressed accordingly to optimize the health status of the patient preoperatively. The patient needed to be highly motivated to undergo surgery and the subsequent rehabilitation. All patients were assessed by the treating team including hand surgeons and physical and occupational therapists. The preoperative assessment included assessment of body functions such as active and passive range of motion, degree of spasticity, grip strength, and perceived pain intensity along with assessment of activities such as grasp ability, activity performance, and occupational performance problems related to upper limb function. All outcome measures have previously been described in detail [13].

#### A.2. Surgical Procedures

The surgical procedures used in this study population were primarily tendon lengthenings and muscle releases. Tenotomy is often done on the tendons of the palmaris longus muscle and the superficial flexor digitorum muscle to the 5^th^ finger. Lengthening a tendon or releasing a muscle from its insertion relaxes the whole muscle-tendon unit. Hence, the spasticity is alleviated but not eliminated. The wrist and the fingers were set in a normal resting position. The tendon lengthening procedure involved a stair-step incision and reattachment in the lengthened position with a side-to-side suture, running cross-stiches. This technique allows for controlled lengthening up to 3 cm, and each tendon attachment can be loaded with 20 kg, which is far more than necessary in daily living tasks.

Suture material was nonresorbable 3-0 Ti-Cron. Resorbable sutures are not recommended due to the long healing time in tendons. With safe sutures, early mobilization on the first postoperative day is possible and recommended to avoid build-up of adhesions. Side-to-side sutures are flat and less bulky than Pulvertaft attachments, allowing for a better cosmetic result.

Muscle release is performed at the insertion site of the pronator teres (PT) and the adductor pollicis (ADP) instead of release at the origin site, which requires a deeper dissection and larger surgery. At tenotomy, the muscle pulls back 2–3 cm (PT) and 1 cm (ADP) and probably stays there to adhere to its surroundings, and a new resting position is found. The muscle still works after surgery but may be weaker. Fractional muscle release is chosen for the brachialis muscle, for instance due to its anatomy. Fractional lengthening cannot be controlled in the same way and usually gives less length. The finger flexors need 3 cm lengthening, and fractional muscle lengthening would add 2 cm and require larger surgery. All the tendons are easily available at the volar distal forearm. The pronator teres may be lengthened if desired.

#### A.3. Postsurgical Treatment

Postoperative care with surgical tape and dressings until the wound is healed is recommended. Early mobilization starting the first postoperative day is usually possible. Meticulous preoperative cautery reduces the risk of bleeding. If there is bleeding due to mobilization, dressing changes are needed and exercises are reduced on the first days. In the study, there were no instances of bleeding that prolonged the rehabilitation time. To prevent postoperative edema and facilitate prolonged soft tissue stretch, wrappings and custom-made orthoses were fashioned the day after surgery. The orthosis was worn around the clock for the first 3 weeks but was removed at training sessions. The training included passive stretching exercises and active dynamic activation of the antagonist muscles, in case of volitional control of those muscles. As a result of the surgical lengthening, the treated muscle was commonly weakened, which increased the patient's potential to voluntarily recruit the antagonists to the spastic muscles. The training started the day after surgery using the concept of early active mobilization to reduce the risk of adhesions, joint stiffness, and muscle weakness. All patients were taught a personalized home training program before discharge. Even though the hand was immobilized in an orthosis, patients were encouraged to use the UL in daily activities to have the muscle pump prevent edema and maintain muscle fitness. The length of stay and postoperative treatment varied depending on the treatment regimen.

All patients returned to the ward three weeks after surgery for follow-up assessments and inpatient rehabilitation. The length of inpatient stay lasted between one and four nights depending on the treatment regimen. Training in daily activities and motor control was now added to the training program, along with tailoring of resting positions. The orthoses were now worn at night only, until at least 3 months after surgery. If needed, the orthosis was readjusted for ideal fit and additional stretch. The continued training was adapted to meet the goals for the individual patient. Follow-up outpatient appointments were scheduled for all patients 3, 6, and 12 months after surgery. The continued training, use of the upper limb in daily activities, and orthosis usage were discussed and tailored to suit the individual patient.
